# Prediction of Ischemic Stroke Recurrence Based on COX Proportional Risk Regression Model and Evaluation of the Effectiveness of Patient Intensive Care Interventions

**DOI:** 10.1155/2022/8392854

**Published:** 2022-06-20

**Authors:** Yun Wang, Ting Lu

**Affiliations:** Department of Neurology Nursing, Sichuan Provincial People's Hospital, University of Electronic Science and Technology of China, Chinese Academy of Sciences Sichuan Translational Medicine Research Hospital, Chengdu, Sichuan 610072, China

## Abstract

With the continuous improvement of medical technology and the aging of the population, the death rate of stroke is gradually decreasing, but the recurrence rate is still high, and the number of recurrences is increasing, resulting in disability and other symptoms, which brings great burden and distress to patients and their families. As the number of strokes increases, neurological impairment becomes more and more severe, affecting patients' ability to live, socialize, and work, and seriously reducing their quality of life. Clustered care is a combination of evidence-based linked interventions and a multidisciplinary team providing the best possible care through evidence-based research and highly operational practice, and it can improve outcomes for ischemic stroke patients more than implementation alone. This paper presents a Cox proportional risk regression-based model, using it to build the most used semi-parametric model for multifactorial survival analysis, due to its advantages of both parametric and nonparametric models, and to analyze the factors influencing survival time in study subjects with incomplete data. The proposed strategy has been found to be useful in predicting ischemic stroke recurrence and cluster care interventions for patients.

## 1. Introduction

Currently, the treatment strategy of ischemic stroke is to improve cerebral blood circulation, restore blood flow in obstructed blood vessels as early as possible, ensure the stability of cerebral blood flow, and reduce neurological damage through pharmacological thrombolysis or mechanical embolization. The advantages, disadvantages, and research progress of cerebral blood circulation improvement therapy, neuroprotective therapy, and preventive therapy for IS are reviewed in order to provide new ideas for the development of IS prevention strategies and therapeutic drugs [1–3].

Irreversible necrosis will develop in the ischemic core area of brain tissue after the development of IS. It is possible to successfully reduce cerebral ischemia damage and recover the structure and function of brain tissue if cerebral blood circulation can be improved promptly within the therapy time window. Measures like thrombus clearance and vasodilation are frequently employed in clinical practice to improve cerebral blood circulation. Within the therapeutic time window, thrombus removal is the most effective way to restore blood flow to the ischemic area. In clinical practice, thrombus removal therapy includes intravenous thrombolysis and endovascular intervention [4–6]. The major thrombolytic method is intravenous thrombolysis using tissue-type fibrinogen activator, which is straightforward, quick, and relatively safe within the therapeutic time window. In addition, neuroprotective agents are a promising IS treatment strategy, which can reduce the extent and degree of neuronal cell death after IS to play an anti-IS role. The main symptoms of ischemic stroke are shown in Figure 1.

Therefore, the clinical translation of neuroprotective agents has become a hot topic of research. The use of tPA beyond the time window (6 h) will lead to an increased risk of hemorrhagic transformation and mortality by four; therefore, only 1% of patients benefit from clinical treatment with t-PA intravenous thrombolysis. There is no significant thrombolytic effect with intravenous thrombolysis for vascular occlusion caused by platelet-rich emboli, old emboli, calcified emboli, or fat emboli. With the maturity of medical imaging technology, scholars found that there exists part of the ischemic semi dark zone with mainly apoptotic neurons in the marginal zone between the normal zone around the central area of ischemia and the ischemic zone, and restoring the blood flow state of the ischemic semi dark zone can stop its transformation into necrotic tissue. Therefore, the brain tissue density and gray-white matter interface of the insular zone after 4.5 h of IS attack were observed with the cooperation of imaging, and patients with small infarct core volume and disproportionate cerebral infarct area were selected for intravenous thrombolytic therapy by assessing the size of salvageable brain tissue. The thrombolytic effect and prognosis were good [7]. One study used CT/magnetic resonance perfusion imaging and RAPID automated software to assess the degree and extent of cerebral ischemia, identify salvageable brain tissue, and screen patients with a perfusion defect-core ischemic area mismatch for t-PA intravenous thrombolysis and showed that good outcomes and prognosis were still achieved by extending the thrombolysis time window to 9 h in the screened patients.

In China, where the nurse-patient ratio is severely imbalanced, targeted evidence-based practice is more conducive to rational deployment of medical resources to improve the quality-of-care delivery in terms of quantity and quality. The development of a clustered nursing intervention program as a link in the distribution of evidence for JBI evidence-based nursing practice integrates evidence into clinical practice in a way that supports nursing interventions' scientific basis in clinical implementation [8, 9]. Clustered care is the construction of specific task lists and standardized care processes. Each care intervention in a structured program is based on high-level clinical evidence, and its effects are greater than the effects of individual interventions through integration, which can be targeted to provide patients with safer and more reliable care and to achieve the best possible outcomes. The single-patient cluster care interventions are not static but are implemented in a way that considers clinical realities and patient wishes. Both patients and caregivers are involved in the health management process, and each intervention is evaluable, providing feedback to clinical staff, improving the quality of clinical care, enhancing the patient-nurse relationship, and increasing patient compliance and satisfaction [10]. Currently, traditional empirical nursing approaches are used to avoid lower extremity DVT in acute ischemic stroke patients, and a scientific preventative system has yet to be developed. The use of mechanical prophylaxis, pharmacological prophylaxis, and early activity alone can improve one aspect of the cause of lower extremity DVT and thus prevent thrombosis, which has been verified in clinical studies. For example, early functional exercise and intermittent pneumatic compression devices can improve the flow rate of blood in patients' lower extremities, accelerate blood flow, avoid blood stagnation in the lower extremities, and prevent the aggregation of clotting factors while through drugs can not only improve the hypercoagulable state of blood, but also increase the risk of bleeding in patients, and how to make the benefits of drug prophylaxis outweigh the risks in patients is still controversial. The occurrence of LDVT is based on high blood viscosity, slow blood flow, and vascular wall. The interconnection and interaction between the three main etiologies of LDVT lead to abnormal clotting of blood to form emboli and impede blood flow. The risk of lower extremity DVT in patients with acute ischemic stroke can be more effectively prevented through the development and implementation of a cluster care intervention program and enhanced health education for patients and caregivers [11].

The Cox proportional risk regression model, also known as Cox regression, was proposed in 1972 and is now the most widely used and classic modelling method in survival analysis. It is primarily used in the medical field for the analysis of prognostic factors in oncology and other chronic diseases, as well as the evaluation of clinical outcomes and etiologic exploration. The application of the Cox proportional risk regression model is limited to some extent by the presence of nonlinear effects between the independent and dependent variables. However, compared with the Kaplan-Meier method, it can satisfy the simultaneous analysis of multiple variables and also analyze the effects of continuous variables on survival outcomes. In this paper, we propose a COX-based proportional risk regression model for ischemic stroke recurrence prediction and patient clustering care intervention.

The paper's organization paragraph is as follows: The related work is presented in Section 2 as well as ischemic stroke disease and bundled patient care.  Section 3 analyzes the methods of the proposed work.  Section 4, discusses the experiments and results. Finally, in Section 5, the research work is concluded.

## 2. Related Work

In this section, we define the ischemic stroke disease, and bundled patient care in depth.

### 2.1. Ischemic Stroke Disease

Stroke is currently the number one disease causing death among Chinese residents. Ischemic strokes account for about 80% of all stroke cases and are characterized by high mortality, disability and recurrence rates, posing a huge burden to the world. Currently, the incidence of ischemic stroke is decreasing year by year in developed countries worldwide, but it is still on the rise in China, making the task of prevention and treatment very difficult. Nerve cells in the brain are highly intolerant to ischemia and hypoxia, and rapid and effective intervention in the acute phase is a key aspect to improve the prognosis of patients with ischemic stroke [12, 13].

The half-life of rt-PA is only 3-5 min, which requires continuous intravenous drip administration, and for strokes caused by acute occlusion of large vessels, the rate of revascularization after rt-PA intravenous thrombolysis does not exceed 25%. Therefore, the search for a drug with a wider therapeutic window, a simpler method of administration (e.g., intravenous push), and a higher revascularization rate has become the goal. The new thrombolytic drugs tenecteplase, a recombinant product, and desmopressin, derived from the saliva of vampire bats, both have higher fibrin specificity and longer half-life than rt-PA; however, whether these drugs are more effective than rt-PA remains to be confirmed in more clinical studies. Endovascular therapy, as opposed to intravenous thrombolytic therapy, provides direct local intervention in thrombosis and theoretically allows for more rapid and effective opening of occluded vessels. Prior to the advent of thrombolytic devices, intra-arterial thrombolysis was used with a view to intervene locally on the thrombus. The ischemic stroke diagnosis process is shown in Figure 2.

The Study of the Use of Recombinant Urokinase Pro in Acute Cerebral Thromboembolism (PROACT)-II has demonstrated that intra-arterial local instillation of urokinase pro has a high rate of revascularization, but with a concomitant increased risk of intracranial hemorrhage. Mechanical thrombolysis relies on local mechanical force to remove the thrombus, theoretically avoiding the effect of drugs on coagulation and thus reducing the risk of bleeding. Mechanical thrombolysis based on intravenous thrombolysis improves the revascularization rate significantly when compared to intravenous thrombolysis alone, while the proportion of patients with 90-day modified Rankin Scale (mRS) scores 0-2 increases significantly, and the risk of bleeding even tends to decrease, demonstrating that thrombolysis [14–16]. Therefore, endovascular therapy is the second breakthrough in the field of ischemic stroke treatment after rt-PA intravenous thrombolysis. Endovascular techniques include intra-arterial thrombolysis and stent retrieval, the latter of which has evolved into thrombus aspiration and Solumbra techniques to further improve recanalization rates, reduce the risk of distal embolism, and mitigate mechanical damage to the cerebral vasculature. Compared with intravenous thrombolysis, thrombectomy has significantly improved the recanalization rate, even up to 90% or more. Further meta-analysis showed that thrombolysis is a highly effective treatment for achieving good clinical outcome, and the treatment time window can be further extended to 7.3 h. For patients with acute occlusion of large cerebral vessels within the thrombolysis time window, bridging therapy remains the gold standard, but it is still controversial whether endovascular treatment should be performed directly instead of intravenous thrombolysis. Some studies suggest that bridging within the time window of thrombolysis is not superior to direct endovascular therapy for ischemic stroke with large vessel occlusion in the anterior circulation, but there are no additional clinical studies to confirm this conclusion [17, 18].

The limited time window for stroke treatment requires that stroke patients be identified and recognized as soon as possible and that emergency systems transport stroke patients to the nearest stroke center as soon as possible. Therefore, it is important to establish a regionalized stroke care network. Primary stroke centers within the network should provide plain-scan computed tomography (CT) and intravenous thrombolysis, while advanced stroke centers should provide more comprehensive neuroimaging, including magnetic resonance imaging, CT angiography, and digital subtraction angiography, with formally trained neurovascular interventionalists, stroke physicians, neurosurgeons, neurologists, and neurocritical care physicians. The mobile CT system allows patients to be seen at the same time. The use of mobile CT allows patients to receive an initial imaging evaluation in the ambulance, while the telemedicine consultation system allows specialists to direct emergency physicians to initiate rt-PA IV thrombolysis prior to transport at any time.

### 2.2. Bundled Patient Care

Bundle of care is a collection of evidence-based interventions offered by a multidisciplinary team using evidence-based research and practice to provide the best possible care, is highly actionable, and can enhance patient outcomes more effectively than if executed separately. The patient cluster care intervention process is shown in Figure 3.

The following factors were generally considered: whether the patient directly benefited, whether the number of days in the hospital was shortened, whether the cost was reduced, and whether the utilization of health care resources was improved. Timely feedback on the results of the implementation of cluster-based care and continuous promotion of its application in clinical practice [19]. Evidence-based care is a nursing concept that has played a huge role in the development of nursing specialization worldwide and has increased as the impact of evidence-based medicine has grown on the medical community. The core idea of evidence-based nursing is the judicious, explicit, and judicious application of the best research evidence to provide the best care for patients with the goal of achieving the best possible recovery outcomes. Evidence-based nursing is primarily a clinical practice based on scientific evidence, combining subjective and objective patient data, clinical experience, and the application of best practice evidence to clinical care and as a basis for clinical care decisions. Cluster-based care is the introduction of evidence-based concepts into clinical practice and the creation of best practice guidelines for the care of patients with prevalent nursing problems or a certain disease, which are highly operational, reliable, and scientific, and their joint interventions are more effective in improving the quality of patient care than individual interventions. The most important feature of clustered care is its ability to integrate with clinical practice, i.e., to apply high-quality evidence that is consistent with clinical scenarios and patient preferences and wishes, thereby promoting the standardization and effectiveness of clinical care practices and improving patient outcomes. In summary, the most important advantage of cluster-based care is that it is based on a combination of patient preferences and clinical scenarios that address the many influencing factors and difficult care issues. Clustered care is supported by evidence-based theory and aims to provide the best and most complete care possible for the patient. It is applied in patients with AIS dysphagia, combining effective interventions and maximizing the impact of each intervention to reduce the incidence of adverse events and improve the patient's recovery outcome. Cluster-based care requires nursing staff to continuously summarize lessons learned and grasp the evidence-based basis when implementing interventions and to give the best care plan based on the original nursing evidence [20, 21].

The concept of clustered care originated from the 1996 to 1998 policy on medical care, stating that evidence-based principles should be followed before all measures are carried out to promote the quality of care. Currently, the international application of clustered care is focused on critical care, emergency care, catheter-associated bloodstream infections, and sepsis, where the rate of catheter-associated bloodstream infections is increasing year by year, accompanied by increased mortality, disability, and length of stay, so clustered care interventions, such as skin preparation with chlorhexidine gluconate, maximizing sterile barriers during placement, selection of subclavian vein placement, hand hygiene, and daily catheterization, which have been categorized by the IHI as central venous catheterization care interventions, have been effective in reducing the incidence of catheter-associated bloodstream infections and improving the quality of life of patients.

## 3. Methods

In the method section, we define the model assumptions and their tests, parameter interpretation, parameter estimation and hypothesis testing, and implementation of a centralized nursing intervention program in detail.

### 3.1. Model Assumptions and their Tests

The COX model recurrence prediction process is shown in Figure 4. The Cox proportional risk regression model is as follows:

(1) $$\begin{array}{c} \text{h}\left(t\right)=h_{0}\left(t\right)\exp\left(\beta_{1}X_{1}+\beta_{2}X_{2}+\cdots +\beta_{P}X_{P}\right). \end{array}$$

From the Cox proportional risk regression model, the ratio of any two individual risk functions, i.e., the risk ratio, is

(2) $$\begin{array}{c} \text{HR}=\frac{h_{i}\left(t\right)}{h_{j}\left(t\right)}=\frac{h_{0}\left(t\right)\exp\left(\beta_{1}X_{i1}+\beta_{2}X_{i2}+\cdots +\beta_{P}X_{iP}\right)}{h_{0}\left(t\right)\exp\left(\beta_{1}X_{j1}+\beta_{2}X_{j2}+\cdots +\beta_{P}X_{jP}\right)}=\exp\left[\beta_{1}\left(X_{i1}-X_{j1}\right)+\beta_{2}\left(X_{i2}-X_{j2}\right)+\cdots +\beta_{p}\left(X_{ip}-X_{jp}\right)\right]\text{i},\text{j}=1,2,\cdots ,\text{n}. \end{array}$$

The ratio is independent of *h*_0_(*t*) and independent of time *t*. That is, the effects of the independent variables in the model do not change with time, and the risk of recurrence for a patient with a particular prognostic factor vector remains in a constant ratio at all-time points to the risk of recurrence for a patient with another particular prognostic factor vector, a situation known as proportional risk. The test for the PH assumption consists of a graphical method and a test method. The graphical method involves observing the distribution or trend of the scattered points in the scatter plot, primarily the COX-KM survival curve, and the graphical method based on the cumulative risk function, the Schoenfeld residual plot, and the Score residual plot to determine whether the survival time satisfies or approximates the PH assumption. The test method is to determine whether the PH assumption is satisfied or approximately satisfied based on the magnitude of the test statistic and the corresponding *p* value, mainly the time covariance method, linear correlation test, weighted residual score test, and the third spline function method. Due to the limitation of space, only the COX-KM survival curve and the graphical method based on the cumulative risk function are introduced here, and readers interested in other methods can refer to the literature.

The COX-KM survival curve method is to observe the Kaplan-Meier survival curves grouped by that variable (meaning the independent variable to be examined), and if the survival curves are significantly crossed, the PH assumption is not satisfied. The graphical method based on the cumulative risk function is to plot the survival curves for each group of the categorical covariate with the survival time *t* as the horizontal axis and the log survival $\ln\left[-\ln\hat{S}\left(t\right)\right]$ as the vertical axis, and the PH assumption is satisfied if the curves corresponding to each group of the covariate are approximately parallel or equidistant. For continuous variables, the variable can be discrete, and the COX-KM survival curves or $\ln\left[-\ln\hat{S}\left(t\right)\right]$ plotted against survival time *t* for each group can be compared, or the interaction term of continuous variables with log survival time can be put into the regression model, and if the interaction term is not statistically significant, the PH assumption is satisfied. If all covariates (meaning independent variables or influences other than time *t*) satisfy or approximately satisfy the PH assumption, the Cox proportional risk regression model can be applied directly.

### 3.2. Parameter Interpretation

Let 8 represent the absolute value of the difference in the value of the *i*^*th*^ independent variable taken on two different individuals, under the condition that the other independent variables take the same value, the variable 8, the natural logarithm of the risk ratio caused by each unit increase *β*in the Cox proportional risk regression model, that is, ln*HR*_*i*_ = *β*_*i*_. When *β* > 0, *HR* > 1, indicating that when *X* increases, the risk function increases, and *X* is risk factor (its real meaning is: such factors take high level relative to take low level risk increase); when *β* < 0, *HR* < 1, it means that when *X* increases, the risk function decreases, and *X* is a protective factor (its real meaning is: such factors take high level relative to take low level risk decrease); when *β* = 0, *HR* = 1, it means that when *X* increases, the risk function remains unchanged, and *X* is a factor with no effect on survival time factors that have no effect on survival time.

### 3.3. Parameter Estimation and Hypothesis Testing

The estimation of the partial regression coefficients *β*_1_, *β*_2_, ⋯, *β*_*p*_ needs to be obtained with the maximum likelihood estimation method with the help of the partial likelihood function. The partial likelihood function is calculated as follows:

(3) $$\begin{array}{c} \text{L}=q_{1}q_{2}\cdots q_{i}\cdots q_{k}=\overset{k}{\underset{i=1}{\prod }}\;q_{i}=\overset{k}{\underset{i=1}{\prod }}\;\frac{\exp\left(\beta_{1}X_{i1}+\beta_{2}X_{i2}+\cdots +\beta_{P}X_{iP}\right)}{\sum_{S\in R\left(t_{i}\right)}\;\exp\left(\beta_{1}X_{s1}+\beta_{2}X_{s2}+\cdots +\beta_{P}X_{sP}\right)}, \end{array}$$

The baseline risk function *h*_*j*_(*t*) in the denominator resists *j* = *i* elimination. Taking the logarithm of the partial likelihood function, the logarithmic partial likelihood function lnL is obtained, and the solution of lnL with the first-order partial derivative of 0 with respect to *β*_*P*_ is obtained (usually a nonlinear iterative algorithm is required, which is omitted here).

The maximum likelihood estimate b of *β* is then obtained. The hypothesis testing approach is comparable to logistic regression analysis, with likelihood ratio test, Wald test, and score test, and the detailed theory is ignored here; both parameter estimation and hypothesis testing may be done quickly with statistical software.

For 0-1 variables (i.e., two-sample survival information), the following expressions hold when the PH assumptions are satisfied:

(4) $$\begin{array}{c} h\left(t\right)=h_{0}\left(t\right)\exp\left(\beta x\right),\\ \begin{array}{c} H\left(t\right)=H_{0}\left(t\right)\exp\left(\beta x\right),\\ \log H\left(t\right)=\log H_{0}\left(t\right)+\beta x\\ \log\left[-\log S\left(t\right)\right]=\log\left[-\log S_{0}\left(t\right)\right]. \end{array} \end{array}$$

For a numerical variable Cox model, the data can be divided into layers based on a numerical variable within the model, and the Cox model is fitted to each layer separately. If the values of each layer are similar to the original model and the plot of log*H*(*t*) or log[−log*S*(*t*)] against t for each layer is approximately parallel, then the risk rate is proportional, and it is appropriate to introduce this variable in the model. This method can also be used for the PH assumption when graphing *k* covariates. Assuming that there are *M* subgroups based on combinations of values of the *k* variables, the *m*-th subgroup will contain individuals with covariate characteristic *X*. The survival curve is estimated within each subgroup by a nonparametric method, i.e., the Kaplan-Meier method, and the *M* groups, can be considered proportional if the plot of the *M* log cumulative risk functions log[−log*S*(*t*)] against *t* is approximately parallel:

(5) $$\begin{array}{c} \hat{w}\left(t\right)=\frac{{\hat{H}}_{1}\left(t\right)}{{\hat{H}}_{0}\left(t\right)}=\exp\left(\hat{\beta }\right),\\ \hat{r}\left(t\right)=\log\left[-\log{\hat{S}}_{1}\left(t\right)\right]-\log\left[-\log{\hat{S}}_{0}\left(t\right)\right]. \end{array}$$

Then, the graph of $\hat{w}\left(t\right)$ or $\hat{r}\left(t\right)$ versus *t* can be used to evaluate whether the PH assumption is satisfied. It is characterized by the evaluation of the constancy of one curve instead of comparing the parallelism of two curves. The scatter plot fluctuates randomly around the center $\exp\left(\hat{\beta }\right)$ or $\hat{\beta }$ under the PH assumption. Note that if *β*(*t*) = log[*h*_1_(*t*)/*h*_0_(*t*)], log[*H*_1_(*t*)/*H*_0_(*t*)] = log[*h*_1_(*t*)/*h*_0_(*t*)] when the PH assumption is satisfied, and not when the PH assumption is satisfied, because log[*H*_1_(*t*)/*H*_0_(*t*)] ≠ log[*h*_1_(*t*)/*h*_0_(*t*)],so *f*(*t*) ≠ *B*(*t*), we cannot infer from (t) from the shape of (1), i.e., such graphs can only give disproportionate baseline risk for each stratum, but not detailed information about the type of deviated risk, which is exactly what we need.

### 3.4. Implementation of a Centralized Nursing Intervention Program

Although DVT prophylaxis has been carried out for many years, it is now commonly believed that DVT occurs mostly in surgical patients, ignoring internal medicine, which lacks awareness of DVT prophylaxis, and even lacks the organizational awareness of multidisciplinary joint DVT prophylaxis. The clinical nursing staff has the most contact time with patients, and the nursing staff has perfect knowledge of thrombosis prevention, which is helpful for early clinical detection of thrombosis risk and prevention. By forming an evidence-based care practice group for prevention of lower extremity DVT in patients with acute ischemic stroke, including evidence-based medical experts, clinical specialists, nursing managers, and nurse specialists, the multidisciplinary team provided a more scientific approach to the construction of the program, increased clinical caregivers' awareness of thrombosis prevention, and ensured the feasibility of the program for clinical research so that patients could receive continuous professional care. The program has improved the awareness of clinical staff on thrombosis prevention, ensured the feasibility of clinical research, and provided patients with continuous professional care.

## 4. Experiments and Results

In this part, we describe the dataset, experimental setup, basic data characteristics, and experimental results in detail.

### 4.1. Dataset

The chronic disease morbidity and mortality surveillance system of a city in China was relied on to construct a cohort of ischemic stroke cases in the city from 2014 to 2018. A total of 16,383 ischemic stroke cases were included according to the International Classification of Diseases criteria for all household residents with stroke established from January 1, 2014, to December 31, 2018, excluding missing or abnormal data.

### 4.2. Experimental Setup

The assessment indexes were measures of vegetation cover, using normalized difference vegetation index (ND-VI), enhanced vegetation index (EVI), and soil adjusted vegetation index (Soi NDVI is the ratio of near-infrared to visible red irradiation, and SAVI is like NDVI with the addition of a soil brightness correction factor). EVI corrects for atmospheric aerosol scattering and soil background based on NDVI and is commonly used in areas with dense vegetation. The values of NDVI, EVI, and SAVI were extracted using ENVI5.3 and ArcGIS10.2 software.

The graph was created using research literature to identify the exposure and result between the intervening factors and to select a minimal set of more appropriate covariates to correct for confounding. According to the DAG plot, age, sex, population density, spatial GDP, walking index, and road density were ultimately selected as the minimum adjusted set on the causal pathway between vegetation cover and stroke death.

Statistical treatment for basic characteristics of the study population, quantitative information was described using (mean ± standard deviation), and qualitative information was described using number of cases and percentages. The Cox proportional risk model was used to quantify the risk ratio of changes in vegetation index to mortality and then adjusted for age, sex, population density, spatial GDP, road density, and walking index. The first quartile (Q1) of NDVI, EVI, and SAVI were used as reference values, respectively, and the 95% confidence interval (CI) of the risk ratio (HR) between quartile (Q2, Q3, Q4) of NDVI, EVI, and SAVI and death from ischemic stroke were reported separately.

### 4.3. Basic Data Characteristics

16383 patients with ischemic stroke and 3697 deaths due to ischemic stroke were included, after quadrating the cumulative mean NDVI, EVI, and SAVI from 2014 to 2018. Among them, 8471 new cases of ischemic stroke in men and 12797 new cases of ischemic stroke ≥60 years old were included.

### 4.4. Experimental Results

The error drop of the model training process is shown in Figure 5. Cox proportional risk regression model analysis of NDVI and risk of recurrence in patients with ischemic stroke quadrupled NDVI and calculated ORs and 95% CIs for Q2 and Q3, using the Q1 group as reference. 1237 deaths from ischemic stroke were recorded in the Q1 group, 843 deaths from ischemic stroke in the Q2 group, 923 deaths from ischemic stroke in the Q3 group, and 694 deaths from ischemic stroke in the Q4. Ischemic stroke claimed the lives of 694 people in the Q4 group. The NDVI-Q4 level was the most protective against death in individuals with ischemic stroke in both the adjusted and unadjusted models for different NDVI levels. In unadjusted model 1, patients with ischemic stroke residing at NDVI-Q4 levels had the lowest risk of recurrence (HR = 0.67, 95% CI: 0.61-0.74), and in model 2, patients with ischemic stroke residing at ND-VI-Q4 levels had the risk of recurrence was lowest in model 2 (HR = 0.67, 95% CI: 0.61-0.73). In model 3, patients with ischemic stroke at the NDVI-Q4 level had the lowest risk of recurrence (HR = 0.63, 95% CI: 0.57 to 0.69) (see Table 1). The performance improvement of the model training process is shown in Figure 6.

Cox proportional risk regression model analysis of EVI and risk of recurrence in patients with ischemic stroke quadrupled the EVI and calculated the OR and 95% CI for Q2 and Q3 using the Q1 group as reference. 1324 deaths from ischemic stroke were recorded in the Q1 group, 818 deaths from ischemic stroke in the Q2 group, 851 deaths from ischemic stroke in the Q3 group, and 851 deaths from ischemic stroke in the Q4 group. The number of deaths from ischemic stroke was 704. In both adjusted and unadjusted models, for different EVI levels, the EVI-Q4 level was the most protective against death in patients with ischemic stroke. In unadjusted model 1, patients with ischemic stroke residing at EVI-Q4 levels had the lowest risk of recurrence (HR = 0.61, 95% CI: 0.55 to 0.66), and in model 2, patients with ischemic stroke residing at EVI-Q4 levels had the lowest risk of recurrence (HR = 0.60, 95% CI: 0.55 to 0.66). The risk of recurrence was lowest in patients with ischemic stroke at the EVI-Q4 level in model 3 (HR = 0.58, 95% CI: 0.53 to 0.63) (see Table 2).

Cox proportional risk regression model analysis of SAVI and the risk of recurrence in patients with ischemic stroke quadrupled SAVI, and the ORs and 95% CIs were calculated for Q2 and Q3 using the Q1 group as a reference. 1108 deaths from ischemic stroke were recorded in the Q1 group, 830 deaths from ischemic stroke in the Q2 group, 915 deaths from ischemic stroke in the Q3 group, and 915 deaths from ischemic stroke in the Q4. The number of deaths from ischemic stroke in the Q4 group was 844. In both adjusted and unadjusted models, for different SAVI levels, SAVI-Q2 levels were the most protective against death in patients with ischemic stroke. In unadjusted model 1, patients with ischemic stroke residing at SAVI-Q2 levels had the lowest risk of recurrence (HR = 0.75, 95% CI: 0.69 to 0.83), and in model 2, patients with ischemic stroke residing at SAVI-Q2 levels had the lowest risk of recurrence (HR = 0.75, 95% CI: 0.68 to 0.83). The risk of recurrence was lowest in patients with ischemic stroke at the SAVI-Q2 level in model 3 (HR = 0.79, 95% CI: 0.72 to 0.86) (see Table 3).

## 5. Conclusion

Clinical utility and extrinsic realism must be considered while evaluating ischemic stroke recurrence prediction models. Clinical usefulness is required for physician approval and use. Firstly, the prediction model should have clinical significance and application value, and secondly, the variables of the model should be easy to collect in the clinical setting, i.e., clinical applicability. Especially for emergency patients or newly admitted patients, good prediction results of the prediction model can guide physicians to make decisions, direct clinical treatment, and secondary prevention and prevent recurrence.

In this study, a hospital-based prospective cohort study was conducted with a 4-year follow-up, and the Cox proportional risk regression model was applied to establish individual equations for ischemic stroke recurrence, and the final variables entered into the main effect equation were as follows: age, heart disease, hypertension, diabetes mellitus, and TC. We also verified the model's external truthfulness, which is one of the most critical requirements for doctors to accept and use it. The established prediction model was initially utilized to forecast the 4-year recurrence rate of ischemic stroke patients, and it has good extrinsic realism and is simple to use with high accuracy, making it ideal for further validation and application promotion.

The construction of a clustered care intervention protocol for lower extremity deep vein thrombosis in patients with ischemic stroke has some clinical applicability and validity. The protocol is based on high-quality evidence, which has changed the status quo of traditional empirical nursing care, promoted the scientific of clinical nursing decisions, ensured the safety of nursing practice, and improved the quality of clinical nursing services. This intensive care intervention program reduces the risk of lower limb deep vein thrombosis in patients with ischemic stroke, improves patients' coagulation function, and facilitates the functional recovery of patients' lower limbs by improving muscle strength, neurological deficits, and functional disability levels, making it clinically valuable.

## Figures and Tables

**Figure 1:** Main symptoms of ischemic stroke.

**Figure 2:** Ischemic stroke diagnostic process.

**Figure 3:** Patient intensive care intervention process.

**Figure 4:** COX model recurrence prediction process.

**Figure 5:** Error drop diagram of model training process.

**Figure 6:** Model training process performance improvement chart.

**Table 1:** Cox proportional risk model analysis of NDVI and risk of recurrence in patients with ischemic stroke.

Models	Quadratic quartiles of NDVI (HR, 95% CI)			
	Q1	95% CI of Q2HR	95% CI of Q3 HR	95% CI of Q4 HR
Model 1	1	0. 68 (0. 63~0. 75)	0.79 (0.72~0.86)	0.67 (0.61~0.74)
Model 2	1	0.68 (0.62~0.74)	0.77 (0.71~0.84)	0.67 (0.61~0.73)
Model 3	1	0. 71 (0. 65~0. 78)	0.74 (0.68~0.81)	0.63 (0. 57~0. 69)

**Table 2:** Results of a Cox proportional risk model analysis of EVI and risk of recurrence in patients with ischemic stroke.

Models	Quadratic quartiles of EVI (HR, 95% CI)			
	Q1	95% CI of Q2HR	95% CI for Q3 HR	95% CI of Q4 HR
Model 1	1	0.64(0.58 to 0.69)	0.69 (0.64~0.76)	0.61 (0. 55~0. 66)
Model 2	1	0. 63(0. 58~0. 69)	0.69 (0.63~0.75)	0.60 (0. 55~0. 66)
Model 3	1	0. 67(0.62~0. 74)	0.67 (0.62~0.73)	0.58 (0. 53~0. 63)

**Table 3:** Results of a Cox proportional risk model analysis of SAVI and risk of recurrence in patients with ischemic stroke.

Models	Quadratic quartiles of SAVI (HR, 95% CI)			
	Q1	95% CI of Q2HR	95% CI for Q3 HR	95% CI of Q4 HR
Model 1	1	0.75 (0.69~0. 83)	0.88 (0. 80~0.96)	0.89 (0.81~0.97)
Model 2	1	0. 75 (0. 68~0. 82)	0.86 (0.79~0.94)	0.88 (0.80~0.96)
Model 3	1	0.79 (0.72~0.86)	0.84 (0.77~0.91)	0.83 (0.76~0.91)

## Data Availability

The datasets used during the current study are available from the corresponding author on reasonable request.
